The article "Artificial Intelligence of Things- (AIoT-) Based Patient Activity Tracking System for Remote Patient Monitoring" was retracted in 2023. Reasons: signs of a paper mill; suspected computer-generated content; unreliable results or conclusions; concerns about the data.

# Artificial Intelligence of Things- (AIoT-) Based Patient Activity Tracking System for Remote Patient Monitoring

**DOI:** 10.1155/2022/8732213

**Published:** 2022-03-01

**Authors:** Timothy Malche, Sumegh Tharewal, Pradeep Kumar Tiwari, Mohamed Yaseen Jabarulla, Abeer Ali Alnuaim, Wesam Atef Hatamleh, Mohammad Aman Ullah

**Affiliations:** ^1^Manipal University Jaipur, Jaipur, India; ^2^School of Computer Science, Dr. Vishwanath Karad MIT World peace University, S. No.124, Paud Road, Kothrud, Pune 411038, Maharashtra, India; ^3^School of Electrical Engineering and Computer Science, Gwangju Institute of Science and Technology, Gwangju, Republic of Korea; ^4^Department of Computer Science and Engineering, College of Applied Studies and Community Services, King Saud University, P.O. BOX 22459, Riyadh 11495, Saudi Arabia; ^5^Department of Computer Science, College of Computer and Information Sciences, King Saud University, P.O. Box 51178, Riyadh 11543, Saudi Arabia; ^6^Department of Computer Science and Engineering, International Islamic University Chittagong, Chittagong, Bangladesh

## Abstract

Telehealth and remote patient monitoring (RPM) have been critical components that have received substantial attention and gained hold since the pandemic's beginning. Telehealth and RPM allow easy access to patient data and help provide high-quality care to patients at a low cost. This article proposes an Intelligent Remote Patient Activity Tracking System system that can monitor patient activities and vitals during those activities based on the attached sensors. An Internet of Things- (IoT-) enabled health monitoring device is designed using machine learning models to track patient's activities such as running, sleeping, walking, and exercising, the vitals during those activities such as body temperature and heart rate, and the patient's breathing pattern during such activities. Machine learning models are used to identify different activities of the patient and analyze the patient's respiratory health during various activities. Currently, the machine learning models are used to detect cough and healthy breathing only. A web application is also designed to track the data uploaded by the proposed devices.

## 1. Introduction

Remote Patient Monitoring (RPM) is an emerging research field that has gained much attention as today's world faces a tremendous need for it in the time of the pandemic. The pandemic has exposed many problems, such as overloading hospitals, the risk of healthcare workers being infected, etc. As a result, there is a need for an RPM system to remotely monitor COVID-negative patients and make the healthcare facility available to COVID-positive patients in the event of an emergency. Even COVID-positive patients can be monitored remotely if they are not in a critical situation. The RPM system assists in remote monitoring in real-time, which enables the detection of specified illnesses rapidly. Using RPM, patients can be monitored from a remote location away from hospital environments using technology. The benefits of using RPM are early detection of patients' health conditions, real-time acquisition of patients' health status, preventing critical health situations, hospitalization, and even deaths.

The article "Artificial Intelligence of Things- (AIoT-) Based Patient Activity Tracking System for Remote Patient Monitoring" was retracted in 2023. Reasons: signs of a paper mill; suspected computer-generated content; unreliable results or conclusions; concerns about the data.

With the help of RPM, medical care services can be provided to patients in case of an emergency. RPM can be implemented for patients with different target groups, for example, patients having chronic illnesses and disabilities, patients with mobility issues, and elderly patients. The primary purpose of RPM is to deliver good healthcare facilities to patients from the comfort of their homes and give them psychological advantages as they are away from the hospital environment. Therefore, the RMP gives patients the freedom and comfort of home and allows them to perform daily activities in their friendly environments while being actively monitored for health conditions. The doctors can also monitor and keep track of patients' health remotely with the help of an automated system capable of generating an alert if something is wrong with the patients' health parameters [1].

To enable such features in the RMP system, this study aims to build a health monitoring device with machine learning (ML) capabilities, network infrastructure, and software applications that will help doctors monitor the activities of their patients and vitals during such activities. Currently, this study focuses on monitoring the activity parameters of patients, such as whether a patient is walking, sleeping, or exercising, and the vitals during these activities, such as heart rate, body temperature, and oxygen level. The novelty of this research is that it uses an edge intelligent decision-making system that immediately identifies the health conditions, suggests patients, and alerts doctors in real-time. Although the proposed approach can analyze only one aspect of RPM, the other parameter for analysis can be easily added to the system, enhancing its capabilities. Therefore, the proposed approach focuses on tracking the patients' activities and different vitals during those activities by implementing the innovative idea to build future intelligent healthcare devices capable of making a decision. The main contributions of this article are as follows:

- An Internet of Things- (IoT-) enabled health monitoring device is designed using the machine learning models to track patient's activities such as running, sleeping, walking, and exercising, the vitals during those activities such as body temperature and heart rate, and patient's breathing pattern during such activities.
- Machine learning models are used to identify different activities of the patient.
- They also analyze the patient's respiratory health during various activities.
- A web application is also designed to track the data uploaded by the proposed devices.

The article "Artificial Intelligence of Things- (AIoT-) Based Patient Activity Tracking System for Remote Patient Monitoring" was retracted in 2023. Reasons: signs of a paper mill; suspected computer-generated content; unreliable results or conclusions; concerns about the data.

The rest of the article can be organized as follows: Section 2 presents the related work.  Section 3 presents the proposed methodology. System architecture is presented in Section 4. Experimental analyses are presented in Section 5.  Section 6 concludes the article.

## 2. Related Work

Nguyen and Silva [2] discussed applications for remotely checking patients for neutralizing cardiovascular illnesses. A telemonitoring system that uses hardware and programming contraptions is proposed by Szydloand Konieczny in [3]. The system is designed to screen diverse heart-related diseases. ECG and heartbeat monitoring system is described in [4] by Lanata et al. In [5], Kozlovszky et al. proposed a method for checking cardiovascular ailments. Blood pressure (BP) and ECG checking systems are discussed in [6] by Ramesh et al. They have developed an algorithm that uses five states. Another approach by Kumar and Kotnana in [7] monitors pulse, heart rate, blood pH level, ECG, and body temperature with the help of different sensors. In [8], Ferreira et al. proposed a system for bedridden patients to monitor ECG, body temperature, oxygen levels, galvanic skin response, and airflow in the lungs. Another approach in [9] proposed by Sannino et al. is used for fall detection of patients using an accelerometer. The system can also monitor other vital signs such as body temperature, oxygen level, ECG, and heart rate. Mishra and Agrawal created a system to collect physiological data for ECG and pulmonary artery pressure (PAP) [10]. The system sends the collected data like text messages. In [11], Pinheiro et al. developed a system for cardiac analysis of a patient in a wheelchair.

Wang et al. in [12] discussed a patient activity monitoring system with fall detection that uses an Android-based Smartphone. Gibson et al. [13] addressed fall detection that uses multiple comparators and a classifier. In [14, 15], a fall detection system is proposed by Paoli et al. and Naranjo-Hernandez et al., which uses a wireless sensor node equipped with an accelerometer and location device. Yu et al. in [16] and Mastorakis and Makris in [17] developed a contactless system based on a camera module for fall detection and physical activity. Greene et al. in [18] developed a method for fall detection based on the Internet of Things (IoT) that uses an Amazon Echo device, a speaker, and a webcam for the functionality.

The article "Artificial Intelligence of Things- (AIoT-) Based Patient Activity Tracking System for Remote Patient Monitoring" was retracted in 2023. Reasons: signs of a paper mill; suspected computer-generated content; unreliable results or conclusions; concerns about the data.

Lanata et al. in [4] proposed a system to monitor patients suffering from mental bipolarity. Nadeem et al. [19] developed a system for EEG signal analysis using Bayesian learning. In [20], Karan et al. proposed a plan to monitor diabetic patients with the help of artificial neural networks. Zhan et al. [21] developed a system called HopkinsPD. This system is designed for patients who are suffering from Parkinson's disease. The system can monitor such patients remotely. Price et al. in [22] developed a system to monitor cognitive fatigue for brain injury people. Prabhakar and Rajaguru proposed the RPM system to classify epilepsy in their study [23]. In [24], Adams et al. proposed another remote patient monitoring system for psychoanalysis. Lakshminarayanan et al. in [25] developed a smartphone-based eye care system that has shown promising results. Rotariu et al. in [26] developed a wireless sensor network-based system for composition and respiration analysis. The system can also analyze melanoma and other skin-related diseases. In [27], Khattak et al. proposed a constrained-oriented application protocol (CoAP) based low-power personal area network system for healthcare. Another application [28] by Gonzalez et al. was developed to assist patients in an accident. Patel et al. in [29] discussed wearable sensors and systems based on microelectromechanical systems (MEMS) and system on a chip (SoC) implementation for rehabilitation applications. Sardini et al. in [30] developed a system using a thin copper wire embedded in a t-shirt with a piezoelectric actuator. The system is used for posture monitoring during rehabilitation. Benelli et al. in [31] proposed a method to measure BP, ECG, body weight, spirometry, and glycemia. A similar approach is proposed in [32] by Sorwar and Hasan to monitor vitals on multiple parameters. E-Ambulance [33] is a system developed by Almadani et al. for remote monitoring of patients. The system is deployed in an ambulance and monitors patients' vital signs while going to the hospital or medical care facility. A Smart Rehabilitation Garment (SRG) for posture correction was developed by Wang et al. [34]. Magno et al. [35] demonstrated a wireless, low-power remote monitoring system with on-body sensors. Serhani et al. [36] created the Smart Mobile End-to-End Monitoring (SME2EM) system for long-term monitoring of disorders that cause illness. The system is deployed as web services and an algorithm to filter and wrapper selection. Al-Naji et al. in [37] developed a camera-based monitoring system to monitor children in a hospital environment. The system monitors respiration rates and detects apnoea using a Kinect camera.

The article "Artificial Intelligence of Things- (AIoT-) Based Patient Activity Tracking System for Remote Patient Monitoring" was retracted in 2023. Reasons: signs of a paper mill; suspected computer-generated content; unreliable results or conclusions; concerns about the data.

Yew et al. [38] proposed an RPM system based on IoT. The system monitors ECG signals and uses the MQTT protocol for data transmission. Annis et al. [39], in their research, studied the RPM system to monitor COVID-19 patients. The system tracks the details of patients based on vitals. Taiwo and Ezugwu [40] also proposed a system to monitor COVID-19 patients. The system is called an intelligent home healthcare support system (ShHeS) and is based on IoT. Iranpak et al. in [41] proposed RMP based on LSTM (long short-term memory) deep neural network algorithm. El-Rashidy et al. in [1] also proposed RPM. The authors have conducted a research survey on principles, trends, and challenges of RPM for chronic disease. These systems are summarized in Table 1. In comparison to the systems described in related works, the proposed system has a novel method of analyzing and monitoring the health parameters of patients, and the proposed system is also extensible as more health parameters can be configured easily.

## 3. Methodology of the Proposed System

Remote patient monitoring (RPM) systems are used to collect various physiological data from patients, which includes electrocardiogram (ECG), body temperature, heart rate, blood oxygen level, blood pressure, respiration rate, and EEG. Various research has been conducted on RPM systems. The proposed system consists of a sensor node to track patients' vitals during different activities which patients perform. The sensor node runs a machine learning model to analyze the vitals during various activities. The sensor node detects the patient's body temperature, heart rate, and oxygen level when the patient is walking, sleeping, or exercising [42, 43]. Analyzing vitals during various activities is critical because these vitals are different during various activities. Thus, by analyzing the vitals during different activities, the doctor can prescribe treatment or give suggestions to patients. For example, if the heart rate is higher during exercise, the doctor may advise the patient or prescribe therapy. Similarly, if the doctor has advised a patient to do some exercise regularly, the doctor can track whether the patient is doing it. Therefore, the proposed solution is helpful for doctors and patients. The doctor can track whether the patient is taking proper rest and exercising daily; on the other hand, patients get health information and alerts if there is a critical situation.

The proposed sensor node collects patients' data using the sensors attached to the nRF5340 Development Kit (DK). The connected sensors are accelerometer, microphone, pulse oximeter, heart rate sensor, and temperature sensor. The accelerometer enables monitoring different patient physical activities, including walking, sleeping, exercising, and running. All these various activities of a patient are identified using the ML model. ML model runs locally on the device and can classify all these patients' activities accurately. With the help of a microphone, the patient's respiratory health can be analyzed. The classification of the patient's respiratory health is also done with the help of an ML model running on the sensor node. The study “Artificial intelligence model detects asymptomatic Covid-19 infections through cell phone recorded coughs” by MIT [44] and research paper “COVID-19 Artificial Intelligence Diagnosis Using Only Cough Recordings” [45] show that this technique is beneficial in detecting the infections. The proposed system uses the Mel Frequency Cepstral Coefficients (MFCC) [46, 47] approach to extract features from the patient's speech signal and compare it with the existing COVID-19 and other sound data available in the database.

The article "Artificial Intelligence of Things- (AIoT-) Based Patient Activity Tracking System for Remote Patient Monitoring" was retracted in 2023. Reasons: signs of a paper mill; suspected computer-generated content; unreliable results or conclusions; concerns about the data.

The study uses two ML models for identifying physical activities and respiratory health. The results of these ML models are programmatically aligned with the results of other sensors such as the pulse oximeter, heart rate sensor, and body temperature sensor to give an overall report of patients' health conditions. For example, when a patient is exercising, the temperature, heart rate, and pulse data may be different from the data acquired while a patient is sleeping. The sensor node also continuously captures the patient's respiratory data via a microphone and detects any anomaly in the respiratory health, such as whether the patient is breathing normally, breathing fast, or having a frequent cough. All these data enable a further study on a different aspect of a patient's health. Figures 1 and 2 depict the other components of the sensor node.

Table 2 contains the list of essential hardware components used for developing the system prototype.

## 4. System Architecture

In the proposed system, the sensor node captures the oxygen level, heart rate, and temperature of patients during different physical activities. This information helps the doctors to study different health parameters based on the activities performed by patients. Along with the physical activities, the sensor node also monitors the respiratory health of the patient. Respiratory health is analyzed while the patient is breathing or making vocal sounds during different activities. The microphone attached to the sensor node is used to capture data for respiratory health analysis. One outcome of the analysis of respiratory health is to detect whether the patient is breathing normally or fast or having a cough. By respiratory analysis using vocal sounds, other conditions such as pneumonia can also be detected.

The article "Artificial Intelligence of Things- (AIoT-) Based Patient Activity Tracking System for Remote Patient Monitoring" was retracted in 2023. Reasons: signs of a paper mill; suspected computer-generated content; unreliable results or conclusions; concerns about the data.

The system works by collecting the data from a sensor node and sending them to the gateway node via Bluetooth or Zigbee. The gateway is present at the patient's sight and displays the result of the analysis by the sensor node. The gateway forwards the data to IoT cloud via Message Queue Telemetry Transport (MQTT) protocol. The data are stored in cloud and can be accessed by the doctors in the dashboard of the web application.  Figure 3 illustrates the overall system architecture.

Figure 4 depicts the sensor node and gateway node prototype. The gateway node is built using Raspberry Pi 3 (RPi3). The RPi3 has built-in Bluetooth Low Energy (BLE), which is used to communicate with the sensor node. The gateway node displays the health information to the patient locally and transmits the data to the IoT cloud server via the MQTT protocol. The gateway node also stores the most recent data in the local database. Once the new readings have been received, the gateway node deletes the previous data, thus making space for more data. Therefore, the gateway node only keeps the current data in a local database, which will be displayed to the patient locally. If patients wish to see historical data, they may use the web application and fetch data from the remote server.  Figure 5 shows the application dashboard.

## 5. Results and Discussion

The proposed system works on two machine learning models: voice data and physical activity data. The proposed method uses Audio Mel Frequency Cepstral Coefficients (MFCC) to extract features from the audio signals for voice data. Edge Impulse TinyML Tool [48] is used to build the proposed model. Tables 3 and 4 show the parameters and cepstral coefficients used for MFCC.

Currently, the ML model predicts two labels for respiratory health that are negative and positive. Negative here means that the patient has healthy breathing. Positive means that the patient has some sort of respiratory sicknesses, such as a cough. The main aim is to detect COVID-19 and pneumonia-positive patients, but the model could not be built due to the unavailability of many audio datasets. The future scope will be the process of collecting the dataset and detecting COVID-19 positive and pneumonia patients.  Table 5 shows the different settings used for training the model.

The neural network architecture for the respiratory health model is given in Figure 6. It consists of an input layer having 650 features, a hidden layer, and an output layer with 2 features. The hidden layer has reshaped layer (13 columns), 1 *D* convolutional/pool layer (8 neurons, 3 kernels, and 1 layer), dropout layer (rate 0.25) for more details refer to [49, 50].

The article "Artificial Intelligence of Things- (AIoT-) Based Patient Activity Tracking System for Remote Patient Monitoring" was retracted in 2023. Reasons: signs of a paper mill; suspected computer-generated content; unreliable results or conclusions; concerns about the data.

Tables 6 and 7 show the training performance of the model. The model is working accurately while being tested on the sample data. As shown in Table 6, the accuracy of a model during training is 100%.

The confusion matrix of the model is as follows.

The result of the live classification is represented in Table 8. In the obtained results, it has been observed that the model can predict cough and healthy breathing with 100% accuracy. Table 8 shows how the model is performing during the live classification for the negative and positive labels at different time stamps.

The second model, which was developed for the proposed system, works on physical activity data. The patient's physical activity data are collected using the 3-axis accelerometer sensor. Currently, the model is trained and tested on four physical activities: exercising, sleeping, running, and stationary. The model works using spectral analysis, which is excellent for analyzing motions. The frequency and power characteristics of a signal over time are extracted from the data collected using input axes *X*, *Y*, and *Z* of the accelerometer. Then, the learning block for classification using Keras [51, 52] has been applied, which helps to learn patterns from data. Anomaly Detection using K-means [53–55] is also used to find outliers in new data. This enables the recognition of unknown states and complements classifiers.  Table 9 shows the parameters of the spectral feature used in the model, which is scaling, filter, and spectral power. The frequency domain and spectral power are represented in Figures 7(a) and 7(b), respectively.

The architecture of the neural network (NN) has been illustrated in Figure 8. NN consists of an input layer with 33 features, hidden layers, and an output layer with four attributes. The hidden layer consists of two dense layers of 20 and 10 neurons, respectively. The training settings are given in Tables 10–12.

The training settings to train the model are provided in Table 10. The parameters used are some training cycles, learning rate, and minimum confidence rating.

The training performance of the ML model for physical activity is given in Table 11, which indicates that the model is performing accurately.

The confusion matrix of the model is given in Table 12. Currently, the model uses four labels that are exercising, moving, running, and stationary. *F*1 score for each label is also given.

The article "Artificial Intelligence of Things- (AIoT-) Based Patient Activity Tracking System for Remote Patient Monitoring" was retracted in 2023. Reasons: signs of a paper mill; suspected computer-generated content; unreliable results or conclusions; concerns about the data.

Figure 9(a) depicts the feature explorer for the model. It is observed that the model can predict each label accurately. Each label in the graphical representation in Figure 9(a) can be clearly seen.

After the live classification, the obtained results are represented in Figures 9(b) and 9(c). Figure 9(b) shows the anomaly explorer. Figure 9(c) shows spectral features from the live classification. The live classification for the “moving” label is shown in Figures 9(b) and 9(c). It is proved that there is no anomaly while classifying data for the moving label. Similarly, from Figure 9(c), it is proved that the model is classifying the moving label accurately.

Table 12 contains a few sample rows of data from the live classification that show that the model is classifying the “moving” label accurately.  Table 13 shows that at a different timestamp, the moving label is classified accurately among all four labels during the live classification of data and no anomaly in the data has occurred.

Similarly, Figures 9(d), 10(a), and 10(b) and Tables 14–16 depict the results from the live classification of accelerometer data for the labels “stationary,” “exercising,” and “running,” respectively. These figures and table data show that like the moving label, the model is also classifying the other three labels “stationary,” “exercising,” and “running” accurately and no anomaly has occurred while classifying the data.

Table 17 and Figure 10(c) show the overall performance of the model developed for the physical activity analysis of the patient.

Figure 11 shows the workflow of the models. As discussed in the previous section, the two models have been developed. For the respiratory health model, the audio data have been fed, which are processed using MFCC. The accelerometer data have been provided for the physical activity model, which are analyzed using spectral analysis.

## 6. Conclusion

An Internet of Things- (IoT-) enabled health monitoring device was designed using the machine learning models to track patient's activities such as running, sleeping, walking, and exercising, different vitals during these activities such as body temperature and heart rate, and patient's breathing pattern during such activities. Machine learning models were used to identify different activities of the patient. Currently, the machine learning models are used to detect cough and healthy breathing only. A web application was also designed to track the data uploaded by the proposed devices. The proposed health monitoring device developed in this study did not cause any discomfort to the patient. It can be easily removed and worn again whenever required without any assistance. The obtained results revealed that the proposed system can be very helpful in monitoring the patients remotely. In the near future, we will extend the proposed device for other kinds of diseases. Additionally, in this article, no machine learning model is proposed. Therefore, we will try to design our own lightweight machine learning model to obtain better results.

The article "Artificial Intelligence of Things- (AIoT-) Based Patient Activity Tracking System for Remote Patient Monitoring" was retracted in 2023. Reasons: signs of a paper mill; suspected computer-generated content; unreliable results or conclusions; concerns about the data.

## Figures and Tables

**Figure 1:** Proposed sensor node.

**Figure 2:** Block diagram of sensor node.

**Figure 3:** System architecture.

**Figure 4:** Nodes: (a), (b), and (c) sensor nodes and (d) gateway node.

**Figure 5:** Application dashboard.

**Figure 6:** Neural network architecture for voice data.

**Figure 7:** (a) Frequency domain (accelerometer data) and (b) spectral power (accelerometer data).

**Figure 8:** Neural network architecture for physical activity model.

**Figure 9:** (a) Feature explorer (physical activity model), (b) anomaly explorer (physical activity model), (c) spectral features (3,001 samples) for *X*-, *Y*-, and *Z*-axis (“moving” label), and (d) spectral features (3,001 samples) for *X*-, *Y*-, and *Z*-axis (“stationary” label).

**Figure 10:** (a) Spectral features (3,001 samples) for *X*-, *Y*-, and *Z*-axis (“exercising” label), (b) spectral features (3,001 samples) for *X*-, *Y*-, and *Z*-axis (“running” label), and (c) testing results for physical activity model.

**Figure 11:** Workflow of the model.

**Table 1:** Summary of the related works.

Authors	Application area	AI-enabled?
Nguyen and Silva [2]	Cardiovascular illnesses monitoring	No
Szydlo and Konieczny in [3]	Heart-related diseases monitoring	No
Lanata et al. in [4], and Kozlovszky et al. [5]	Cardiovascular ailments analysis	No
Ramesh et al. [6]	Blood pressure (BP) and ECG monitoring	No
Kumar and Kotnana [7]	Pulse, heart rate, blood pH level, ECG, and body temperature monitoring	No
Ferreira et al. [8]	Monitor ECG, body temperature, oxygen levels, galvanic skin response, and airflow in the lungs	No
Sannino et al. [9]	Fall detection of patients using an accelerometer, body temperature, oxygen level, ECG, and heart rate monitoring	No
Mishra and Agrawal [10]	ECG and pulmonary artery pressure (PAP) monitoring	No
Wang et al. [12], Gibson et al. [13], Paoli et al. [14], Naranjo-Hernandez et al. [15], Yu et al. [16], Mastorakis and Makris [17], and Greene et al. [18]	Fall detection monitoring	No
Lanata et al. [4]	Mental bipolarity monitoring	No
Nadeem et al. [19]	EEG signal analysis using Bayesian learning monitoring	No
Karan et al. [20]	Monitor diabetic patients with the help of artificial neural networks	No
Zhan et al. [21]	Parkinson's disease monitoring	No
Price et al. [22]	Cognitive fatigue for brain injury monitoring	No
Prabhakar and Rajaguru [23]	Classifying epilepsy	No
Adams et al. [24]	Psychoanalysis monitoring	No
Lakshminarayanan et al. [25]	Eyecare	Yes
Rotariu et al. [26]	Respiration analysis, melanoma, and other skin-related diseases	No
Khattak et al. [27]	Healthcare system	No
Gonzalez et al. [28]	Assist patients in an accident	No
Patel et al. [29]	Rehabilitation applications	No
Sardini et al. [30]	Posture monitoring during rehabilitation	No
Benelli et al. [31]	BP, ECG, body weight, spirometry, and glycemia	No
Sorwar and Hasan [32]	E-health monitoring	No
Almadani et al. [33]	Ambulance and monitors patients' vital signs	No
Wang et al. [34]	Posture correction	No
Magno et al. [35]	On-body sensors for monitoring	No
Serhani et al. [36]	Monitoring of disorders that cause illness	No
Al-Naji et al. [37]	Camera-based monitoring system to monitor children in a hospital environment	No
Yew et al. [38]	ECG monitoring	No
Annis et al. [39] and Taiwo and Ezugwu [40]	Monitor COVID-19 patients	No
Iranpak et al. [41]	General monitoring	Yes
Wang et al. [12]	Disease-based monitoring	Yes

The article "Artificial Intelligence of Things- (AIoT-) Based Patient Activity Tracking System for Remote Patient Monitoring" was retracted in 2023. Reasons: signs of a paper mill; suspected computer-generated content; unreliable results or conclusions; concerns about the data.

**Table 2:** Components of the system.

Hardware components		Description
Processor	nRF5340 Development Kit	It is the brain behind the system. It is an SoC, powered with two-arm® cortex®-M33 processors, has all the processing power to execute machine learning model and built-in communication modules such as BLE, Zigbee, Thread. The kit is used to design sensor nodes.
	Raspberry Pi 4	It has Broadcom BCM2711, quad-core Cortex-A72 (ARM v8) 64-bit SoC @ 1.5 GHz. This kit is used to design gateway nodes for the system.
Sensors	X-NUCLEO-IKS02A1 Shield	It is an industrial motion MEMS sensor expansion board. It embeds the following modules.
		(i) ISM330DHCX 3-axis accelerometer
		(ii) 3-axis gyroscope
		(iii) IIS2MDC 3-axis magnetometer
		(iv) IIS2DLPC 3-axis accelerometer
		(v) IMP34DT05 digital microphone
		The accelerometer and microphone are used in the proposed system.
	SparkFun Digital Temperature Sensor	It is used for reading body temperature.
	SparkFun Pulse Oximeter and Heart Rate Sensor	It is used to monitor patients' heart rate and oxygen saturation.

**Table 3:** MFCC parameters.

Parameter	Value
Number of coefficients	13
Frame length	0.02
Frame stride	0.02
Filter number	32
FFT length	256
Window size	101
Low frequency	300

**Table 4:** Cepstral coefficients.

Parameter	Value
Coefficient	0.98
Shift	1

**Table 5:** Training settings.

Settings	Value
Number of training cycles	100
Learning rate	0.005
Minimum confidence rating	0.60

**Table 6:** Training performance.

Accuracy	Loss
100%	0.00

**Table 7:** Confusion matrix.

	Negative	Positive
Negative	100%	0%
Positive	0%	100%
*F*1 score	1.00	1.00

The article "Artificial Intelligence of Things- (AIoT-) Based Patient Activity Tracking System for Remote Patient Monitoring" was retracted in 2023. Reasons: signs of a paper mill; suspected computer-generated content; unreliable results or conclusions; concerns about the data.

**Table 8:** Live classification (respiratory health model).

Timestamp	Negative	Positive
0	0.25	0.73
500	0.15	0.85
1000	0.04	0.96
1500	0.03	0.97
2000	0.03	0.97
2500	0.08	0.92
3000	0	0.99
3500	0.81	0.19

**Table 9:** Spectral features parameters.

Parameter		Value
Scaling	Scale axis	1
Filter	Type	Low
	Cut off frequency	3
	Order	6
Spectral power	FFT length	128
	No. of peaks	3
	Peaks threshold	0.1
	Power edges	0.1, 0.5, 1.0, 2.0, 5.0

**Table 10:** Training settings.

Parameter	Values
Number of training cycles	100
Learning rate	0.0005
Minimum confidence rating	0.60

**Table 11:** Training performance.

Accuracy	Loss
100.0%	0.00

**Table 12:** Confusion matrix.

	Exercising	Moving	Running	Stationary
Exercising	100%	0%	0%	0%
Moving	0%	100%	0%	0%
Running	0%	0%	100%	0%
Stationary	0%	0%	0%	100%
*F*1 score	1.00	1.00	1.00	1.00

**Table 13:** Live classification (accelerometer data) for “moving” label.

Timestamp p	Exercising	Moving	Running	Stationary	Anomaly
0	0	1.00	0	0	−0.04
80	0	1.00	0	0	−0.05
160	0	1.00	0	0	−0.05
240	0	1.00	0	0	−0.05
320	0	1.00	0	0	−0.05
400	0	1.00	0	0	−0.05
480	0	1.00	0	0	−0.05
560	0	1.00	0	0	−0.05
640	0	1.00	0	0	−0.04

**Table 14:** Live classification (accelerometer data) for “stationary” label.

Timestamp p	Exercising	Moving	Running	Stationary	Anomaly
0	0	0	0	0.99	−0.12
80	0	0	0	0.99	−0.12
160	0	0	0	0.99	−0.12
240	0	0	0	0.99	−0.12
320	0	0	0	0.99	−0.12
400	0	0	0	0.99	−0.12
480	0	0	0	0.99	−0.12
560	0	0	0	0.99	−0.12
640	0	0	0	0.99	−0.12

**Table 15:** Live classification (accelerometer data) for “exercising” label.

Timestamp	Exercising	Moving	Running	Stationary	Anomaly
0	1	0	0	0	0.03
80	1	0	0	0	0.14
160	1	0	0	0	0.12
240	1	0	0	0	0.11
320	1	0	0	0	0.16
400	1	0	0	0	0.15
480	1	0	0	0	0.08
560	1	0	0	0	0.12
640	1	0	0	0	0.12

**Table 16:** Live classification (accelerometer data) for “exercising” label.

Timestamp	Exercising	Moving	Running	Stationary	Anomaly
0	0	0	1	0	−0.11
80	0	0	1	0	−0.27
160	0	0	1	0	−0.2
240	0	0	1	0	−0.22
320	0	0	1	0	−0.1
400	0	0	1	0	−0.06
480	0	0	1	0	−0.17
560	0	0	1	0	−0.14
640	0	0	1	0	−0.12

**Table 17:** Testing analysis for physical activity model.

Exercising	Moving (%)	Running	Stationary (%)	Anomaly (%)
Exercising	99.95	0.05%	0	0
Moving	0.10	99.98%	0.05	0.05
Running	0.01	0.09%	99.9	0
Stationary	0	0.10%	0.05	99.85
*F*1 score	99.90	99.85	99.87	99.95

## Data Availability

The data used to support the findings of this study are available from the corresponding author upon request.
